# Homogeneous Decision Community Extraction Based on End-User Mental Behavior on Social Media

This article has been retracted.

**DOI:** 10.1155/2022/3490860

**Published:** 2022-03-08

**Authors:** Suneet Gupta, Sumit Kumar, Sunil L. Bangare, Shibili Nuhmani, Arnold C. Alguno, Issah Abubakari Samori

**Affiliations:** ^1^Department of CSE, School of Engineering and Technology, Mody University, Lakshmangarh, Rajasthan, India; ^2^Indian Institute of Management, Kozhikode, India; ^3^Department of Information Technology, Sinhgad Academy of Engineering, Savitribai Phule Pune University, Pune, India; ^4^Department of Physical Therapy, Imam Abdulrahman Bin Faisal University, Dammam, Saudi Arabia; ^5^Department of Physics, Mindanao State University, Iligan Institute of Technology, Tibanga Highway, Iligan, Philippines; ^6^School of Engineering Sciences, University of Ghana, Accra, Ghana

## Abstract

Aiming at the inadequacy of the group decision-making method with the current attribute value as interval language information, an interval binary semantic decision-making method is proposed, which considers the decision maker's psychological behavior. The scope of this research is that this paper is based on localized amplification method. The localized amplification method used in this research may amplify physiological movement after removing unwanted noise, allowing the movement trend to be seen with the naked eye, improving the CNN network's mental identification accuracy. These two algorithms analyze the input picture from various perspectives, allowing the CNN network to extract more information and enhance identification accuracy. A new distance formula with interval binary semantics closer to decision-makers thinking habits is defined; time degree is introduced. An optimization model is established to solve the time series weights by considering the comprehensive consistency of expert evaluation. Based on prospect theory, a prospect deviation value is constructed and minimized weight optimization model, using the interactive multiple attribute decision community making (TODIM) method based on the new distance measure to calculate the total overall dominance of the schemes to rank the schemes. Taking the selection and evaluation of supply chain collaboration partners as an example, the effectiveness and rationality of the proposed method are verified.

## 1. Introduction

With the increasing complexity of decision-making problems in various fields, individual decision-making has long been unable to meet the requirements of scientific decision-making, and group decision-making has attracted more and more attention and attention from experts and scholars [1, 2]. For multiattribute group decision-making, most existing research is based on the classical expected utility theory, which assumes that the decision-maker is entirely rational, but this is not in line with reality. Prospect theory [3, 4] believes that decision-makers have systematic perception bias in the decision-making process. Decision-makers do not continuously pursue the maximum utility in behavior but show reference dependence and loss aversion. Therefore, it is necessary to consider the psychological behavior of decision community makers in the decision-making process.

In addition, in the entire group decision-making process, due to the limitations of gender and decision makers' cognition, decision-makers are more inclined to give evaluations in natural language. [5] proposed a binary semantic information evaluation model, which attracted the attention of scholars at home and abroad. At present, the research based on binary semantics mainly focuses on two aspects: on the one hand, the research on binary semantics set counters [6–10]. However, in the actual decision-making process, due to the ambiguity of decision-making information and the limitations of decision-makers cognition, decision-makers are often more willing to give evaluation information in the form of interval language to reduce decision-making pressure. In response to such problems, [11] showed the definition of interval binary semantics and several set counters and used the interval binary semantic possibility formula to sort the solutions; reference [12], based on the maximum dispersion [13], defined a new interval binary semantic Bonferroni average operator and its corresponding weighting method; reference [14] combined interval binary semantics and VIKOR method, and proposed an outsourcing supplier selection method; reference [15] proposed a subway door failure risk assessment method based on interval binary semantics and failure mode. The method proposed in the literature [11–15] has the following shortcomings: first, the evaluation information is uniformly distributed in the interval by default, and the distribution of information in the gap that is more in line with the psychology of decision-makers is not considered; second, most of the existing research in the single static stage, [16] it is not suitable for the situation that requires dynamic multistage analysis; thirdly, the above methods all assume that the decision-maker is entirely rational, [17] but in the actual decision-making, the decision-makers psychological behavior is often bounded rationality. The impact of social media on mental health is stress, anxiety, and sadness which have all been related to the social network use. Individuals who often use digital platforms, according to latest studies cited by The Young Mind Centre and The National Centre for Health Research, are more sad and unhappy with life than others who stay longer on nonscreen-related activities. To sum up, based on existing research, this paper proposes an interval binary semantic dynamic group decision-making that considers the decision maker's psychological behavior for the multiattribute group decision-making problem in which the attribute value is interval language, and the attribute weight and time series weight are entirely unknown method. Considering the thinking habits of human beings, it is believed that the density of evaluation information in the interval is more similar to the normal distribution, and based on this, a new interval binary semantic distance formula is proposed. Solve the time series weights based on the time degree and entropy; [18, 19] by determining the positive ideal scheme under each time series, establish a prospect theoretical profit and loss matrix, and build a linear programming model to minimize the sum of the squares of the foreground deviation values, and determine the attribute weights under each time series; then, Construct an ITL-TODIM method based on interval binary semantic distance measure to calculate the complete overall dominance of each candidate scheme, and determine the pros and cons of the system according to the total general authority; the evaluation is used as an example to verify the effectiveness and rationality of the proposed method. The ITL-TODIM approach which is based on intermediate binary semantic distance measure to compute the total overall dominance of each candidate scheme and identify the system's advantages and disadvantages in terms of total general authority. The evaluation is used as an example to check the suggested method's efficacy and reasonableness. The TODIM technique completely analyses managements' risk aversion perspective and may represent key stakeholders' risk preference by altering the dimensions, which is more in accordance with the actual decision-making needs. Any two possibilities, however, must be evaluated using the TODIM approach, which has a significant computational cost. Psychological behavior is one of the main ways people express their emotions. Research on various expression recognitions has made significant progress [1–6]. In recent years, the recognition of spontaneous expressions has become a new research hotspot [7, 8], and psychological expressions are often generated when people want to suppress their feelings, which can neither be faked nor suppressed [7–9]. The complete expression usually lasts 0.5∼4 s [10], which is relatively easy to be recognized by people. However, psychology believes that when a person tries to hide his genuine emotions, occasionally, there are emotions that leak out. Psychological behaviors were first discovered in 1966 [20]. Three years later, [21] used the term psychological behaviors when analyzing a video interview of a patient who attempted suicide. Psychological behaviors usually change uncontrollably between 1/25 and 1/2 s [22], and the frequency of occurrence is low, and untrained individuals do not have high recognition ability [23]. Therefore, the results reported by different researchers also vary considerably [11, 24]. After this, Ekman and Friesen proposed the Brief Affect Recognition Test (BART) in 1979 [12]. In subsequent experiments, they found that the subjects' psychological-expression recognition ability was positively correlated with lie recognition ability [13]. Afterwards, the Japanese and Caucasian Brief Affect Recognition Test (JACBART) [14, 15] was conducted, verifying that the subjects' psychological-expression recognition ability was positively correlated with lie recognition ability [20], it can be proved that psychological-expressions can effectively help people identify lies. Face psychological expression recognition involves image processing and analysis, computer vision, artificial intelligence, psychology, biology, and other directions.

## 2. Literature Survey

In 2002, Authors [24] developed a psychological-expression recognition tool, METT (Psychological behavior Training Tool). Studies have shown that METT tools can improve an individual's ability to recognize psychological expressions by 30% to 40% on average. In addition, an Action Coding System (FACS) [21] is also designed, according to the anatomical characteristics of the face, it is divided into several independent and interconnected motion units (Action Unit, AU), The motion characteristics of these motor units and the main areas they control and the expressions associated with them are analyzed, and a lot of photo descriptions are given. Although human emotions are complex and diverse, they can still be divided into 6 basic emotional categories [22, 23]. Therefore, researchers combine different motor units to form FACS codes to correspond to different expressions, mainly divided into happy, angry, fearful, sad, surprised, and others. When people express their inner state and psychological needs, they will produce many psychological behaviors [24]. Still, because psychological expressions exist for too short a time and are not easily detected by the human eye, computers can be used to solve this problem.

## 3. Psychological-Expression Recognition Technology

Psychological expression is the tiny movement change of the human face, including texture change. The movements of psychological expressions are too small and of short duration to be easily captured by the human eye. The physical character of all substances is dictated by their real physical composition, which is referred to as texture. Textures can elicit behavioral processes in people. This mental reaction enables us to feel something without really touching it. The blood circulation in our faces alters as we experience various emotions. This causes tiny colour shifts that other persons might see. People can properly determine someone's sentiments from these visual shifts up to 75% of the time, according to recent research. Therefore, the psychological expressions of the face can be studied through machine vision. According to the above characteristics, several mainstream methods for psychological-expression recognition are Convolution Neural Networks (CNN) [11], Optical Flow (Optical Flow) method, and Local Binary Pattern (LBP).

### 3.1. Convolution Neural Networks

Convolution Neural Networks (CNN) [11] has been widely used in various fields such as machine vision and speech recognition since their birth. Usually, CNN is used as feature extraction and depth feature extraction for image class input, and the desired output results can be obtained after analyzing the extracted features. Relatively small movements characterize Psychological-expressions. If convolution neural networks are used, it is usually necessary to use other auxiliary methods to change the input of the web, or to change and optimize the network structure so that the network can extract more valuable features, thereby improving the recognition of psychological-expressions accuracy.

### 3.2. Local Binary Patterns and Improvement Methods

Local Binary Patterns (LBP) [12] can effectively deal with illumination changes and are widely used in texture analysis, texture recognition, and other fields, with grey and rotation invariance degeneration and other significant advantages. The LBP value of the central pixel reflects the texture information of the surrounding area of the pixel, as shown in Figure 1.

This feature is widely used because of its simplicity and ease of computation. However, the traditional LBP algorithm cannot be applied to video signals for video images, so some improvements to the LBP algorithm are needed. Among them, [25] proposed a robust dynamic texture descriptor that performs local binary patterns from three orthogonal planes (LBP-TOP), widely used for psychological behavior. To consider both the spatial and temporal information of the video, LBP-TOP extends LBP. Compared to LBP, this method finds three types (*XY*, *XT*, *YT*) instead of one plane (spatial *XY*). Given a video sequence, it can be viewed as a stack of *XY*, *XT*, and *YT* planes along the temporal *T*-axis, spatial *Y*-axis, and spatial *X*-axis, respectively. The three histograms come from three planes, respectively, and are concatenated into one histogram as a dynamic video texture descriptor, as shown in Figure 2. LBP-TOP extends the application of the LBP algorithm to a higher dimension and can identify textures in time series. The information between the frames before and after is correlated through this method, making the LBP algorithm more widely used. Local Binary Patterns (LBP) are frequently employed in texture analysis, texture identification, and other domains and have major benefits such as grayscale and rotation invariance degradation. The texture knowledge of the pixel's surrounding area is reflected in the central pixel's LBP value. Any radius and number of neighborhood pixels may be achieved by using a circular neighborhood and subsection linear interpolation data at noninteger pixel locations. The complimentary comparison measure might be the grey scale variation of the immediate region.

They generate fairly extensive descriptive statistics, which slow down identification speed, particularly on huge face databases. (2) They overlook the spatial patterns in some circumstances because they do not examine the influence of the central pixel.

The properties of LBP can be found in LBP-TOP, and vice versa. LBP-TOP is unaffected if the pixel value increases or lowers by the same amount. This method can be employed in real life despite the interference to the image created by the natural parallel light environment, when in, the robustness is very high. However, because it is pixel-based, this method requires more expertise in Computer Science and Engineering. The first use of LBP is to compare the centre pixel to *P* pixels in the vicinity of radius *R*. When *R* is 1, the centre pixel and the surrounding 8 pixels have a size of 2*P*. The final size is 28 × 256. *R* is no longer a single number, and the size of the neighborhood grows exponentially. The LBP operator's mode type is utilized for dimensionality reduction in [26]'s proposal to employ a “equivalent pattern” (Uniform Pattern) as a solution to this problem. There are two transitions from 0 to 1 or 0 to 1, according to Ojala et al., in natural images. As a result, the “equivalent mode” is defined as having at most two transitions from 0 to 1 or 1 to 0 in a cyclic binary integer. An analogous Pattern class refers to the binary that corresponds to the LBP. It takes 256 to get down to 58 using this strategy. In other words, the values are divided into 59 categories, with the 58 uniform patterns constituting one and the remaining values constituting the 59th. Consequently, the histogram's 256-dimensional dimension is reduced to 59 dimensions using this method, rather than the original 2*P*'s *P* (*P* − 1) + 2. This decreases the influence of high-frequency noise on the eigenvectors by making them less dimensional. Using LBP-TOP, an image is divided into 59 × 3 blocks, with each block generating an array with a size of 3.59. This is because LBP-TOP applies LBP in the time dimension. The finished feature's dimensions are 4 × 4 × 59 × 3 = 2.832. LBP-TOP is a high-dimensional characteristic that has a significant impact on calculation speed and accuracy.

## 4. Mental Behavior for Psychological Change

Psychological-expression recognition has made some progress at present, but there is still a lot of room for improvement in technology. The following is an analysis and prospect of the problems existing in different methods of psychological expression:

- Convolution neural network used as a Traditional method is widely used, and the current mainstream idea is to use the optical flow method as input and combine it with LSTM to achieve better results. However, there is a fatal problem in using convolution not high. For convolution neural networks, it is a small sample problem. Therefore, data enhancement is required during calculation, or Cross-domain experiments, while improving robustness. In the subsequent process, you can try to use transfer learning, which can alleviate the problem of overfitting to a certain extent. In addition, you can also use methods such as adversarial neural networks to generate some samples for training, which can alleviate the problem of small sample data.
- There are three main methods of feature screening: filter, wrapper, and embedded. The filtering feature selection method assigns weights to the features of each dimension, and then sorts the features according to the weight; the encapsulating feature selection method views subset selection as an optimization problem, generates different combinations, evaluates the combinations, and then compares them with others. By comparing the two approaches, we can determine which features are most critical for a specific model to be trained with. There are three basic screening procedures, and each is designed for a certain scenario. The statistical performance of all training samples is directly used to evaluate the relevance of each feature in the filtering feature selection technique. Although its performance is excellent, this algorithm has a lot of advantages, including the ability to remove a large number of unnecessary attributes, its universality, and the ability to prescreen features. It is necessary to combine the feature selection approach with the subsequent classification algorithm, evaluate each feature's significance based on the classifier's accuracy, and select the ideal feature subset for a certain classification algorithm. It is similar to the filtering approach, but the integrated feature screening method uses machine learning training rather than relying solely on the statistical indications of a feature to evaluate its advantages and disadvantages. Machine learning is also used in the embedding method, as opposed to the packaging method. With this approach, all of the features are used for training, rather than just a subset of them. By utilizing the embedded feature selection method, both the feature selection and learner training are done in the same optimization process. Each of the three ways has its own pros and weaknesses; therefore they can all be utilized together. An ideal subset of features is picked out based on preprocessing and classifier approach advantages in order to increase the accuracy of psychological-expression recognition.

## 5. Psychological-Expression Recognition Method

### 5.1. Method  for Psychological-Expression Recognition Based on CNN

CNN is a commonly used method when processing image signals. Still, because the psychological-expression changes are relatively small, the effect of only using CNN is not very good, so some literature choose to process the input image. The traditional psychological-expression feature extraction needs to consider the spatial image features and the temporal sequence. The amount of pixels used to generate a digital image is referred to as spatial resolution. Higher spatial resolution images include more pixels than lower spatial resolution images. Object (matrix) and picture (graph) modes are available for representing spatial objects. Each spatial object can be specified as a spot, line, or polygon in object mode. Each spatial object can be specified in picture mode as a collection of adjacent cells called regions. Generally, feature extraction is performed on all frames of the psychological expression from the beginning to the end, while proposng a psychological expression. Stage classifier: First, the psychological expressions are divided into three stages: onset, peak, and offset using temporal information, and then spatial information is used to detect intensity changes. Compared with the traditional psychological-expression feature extraction method, this method only uses a psychological-expression (Apex) frame and an initial (Onset) frame to extract features, increasing the number of valid frames reducing the amount of computation and outperforms other traditional methods. In addition, [30] proposed a video magnification method based on eye interference elimination and used convolution neural network to realize the task of psychological-expression recognition. First, zoom in on the data to extract the eye position coordinates. After that, the original eye video will be replaced with the enlarged video for image fusion to eliminate eye interference. Finally, the convolution neural network model network is designed using the idea of VGG16 to realize emotion recognition. The local amplification technology applied in this paper can amplify the psychological-expression movement after reducing the noise interference so that the movement trend can be seen by the naked eye, which can increase the accuracy of the CNN network for psychological-expression recognition. These two methods process the input image from different angles so that the CNN network can better extract features and improve the accuracy of recognition. They generate fairly extensive descriptive statistics, which slow down identification speed, particularly on huge face databases. (2) They overlook the spatial patterns in some circumstances because they do not examine the influence of the central pixel.

At present, most of the psychological-expression feature extraction based on CNN is combined with the optical flow method extraction, which is also one of the advantages of the CNN framework. However, if CNN is used for deep learning, it is still unrealistic for the current data set. The amount of data in the existing data sets cannot meet the needs of the deep learning network, and it is easy to cause overfitting, which leads to the huge size of CNN. The advantage cannot be played.

### 5.2. Psychological-Expression Recognition Method Based on Optical Flow Method

FACS requires motion records of various positions such as eyebrows and mouth corners as an essential tool for recognizing psychological expressions. This method uses ROIS and HOOF features together, and the obtained results correspond to AU, which can identify psychological expressions more accurately. Psychological-expression detection is often independent, and a long-video expression automatic recognition method consisting of macros and psychological expressions (time segmentation). This method utilizes the stress generated by nonrigid motion on the skin during the expression process. It uses the central difference method to calculate the solid and dense optical flow field observed in several areas of each subject's face (chin, mouth, cheeks, forehead). Strain level: This method can successfully detect and distinguish psychological expressions and fast local psychological expressions, which is of great help to the detection of psychological expressions in complex scenes.

### 5.3. Method of Psychological-Expression Recognition

According to the problems of LBP-TOP, STCLQP adds information such as amplitude and direction components, extracts more helpful information, and fuses the extracted data into a feature vector, which improves the utilization of image features. Compared with LBPTOP, the STCLQP method extracts more information and thus results in higher dimensionality. In this paper, the LQP technique is used. Compared with the LBP, whose dimension increases exponentially with the neighborhood radius *R*, LQP maps the extracted features to the lookup table. When *R* increases, the dimension no longer shows exponential growth. Therefore, this method is more suitable when the *R*-value needs to be improved, and because the LQP technology alleviates some of the previously extracted more dimensional information.

LBP-SIP reduces redundancy in LBP-TOP mode, provides a more compact and lightweight representation, improves accuracy, and reduces computational complexity. Unlike LBP-TOP, this method only uses 4 pixels at the top, bottom, left, and right of a pixel at time *t* and 6 pixels at the same position at time *t* − 1 and *t* + 1. Because the extracted features are few, it is more suitable when there are many images and a long time, and the operation is faster than LBP-TOP. Its speed is 2.8 times that of LBPTOP. The feature extraction time of this method is 15.88 s, which is about 2.4 s faster than that of the LBPTOP method, and the recognition time is 0.208 s, which is 0.3 s more quickly than the LBP-TOP method. Compared with the LBP-TOP method, LBP-SIP reduces a considerable amount of time, but this time is still too long for subsequent practical applications to achieve real-time detection. But it provides an idea to reduce the processing time. In addition, to reduce the dimension of the features extracted by LBP-TOP and then use SVM for classification. This method first uses the LBP-TOP operator to extract psychological-expression features. It then proposes a feature selection algorithm based on Relief combined with a Locally Linear embedded (LLE) manifold learning algorithm, which can effectively reduce the number of postextraction features. Feature dimension: Finally, the SVM classifier with Radial Basis Function (RBF) kernel is used for classification, and good results are obtained. This method is based on the LBP-TOP method for feature vector extraction, so the application environment is consistent with LBP-TOP. The filter method is used to exclude irrelevant features, and then the wrapper method is used to filter out the features with greater influence, which avoids the dimensional disaster and reduces the amount of calculation accordingly. This method gives a direction for future development. It is a revelation that for the pixel-by-pixel feature extraction method of LBP-TOP, the extracted features can be screened to improve the recognition accuracy during classification.

For the redundant features of LBP-TOP, the above methods adopt different ideas for dimensionality reduction, but it is far from enough for practical application in real life. The method of pixel-by-pixel feature extraction is easy to cause dimensional disasters. The selection of features and feature extraction methods is particularly important before. It is only when the processing speed is reduced that there is an opportunity to apply such methods to social life.

#### 5.3.1. CNN (Convolution Neural Network)

CNN is an excellent method for dealing with image problems, but the network structure needs to be adjusted for different issues. When using CNN, feature extraction is usually performed first, and then further processing is performed after the features are extracted. However, the optical flow method and the improved local binary mode method use different removal methods. For the feature map, CNN can continue to extract deep features, so the use of CNN and optical flow method and local binary mode improvement method does not conflict with itself. CNNs are often used in conjunction with a popular form of recurrent neural network called the Long Short-Term Memory (LSTM) module for video-type files.

#### 5.3.2. Applicable Scene Analysis of CNN

Optical flow method and improved local binary mode of the existing psychological-expression recognition methods are all based on datasets. The generalization ability of psychological-expression recognition, in reality, is not high and cannot be applied. However, the required environment and application scenarios can be estimated according to the characteristics of existing methods. As far as the current development is concerned, if the multiple existing networks are integrated into the detection of psychological-expression recognition, complex scenes can be detected, such as shopping malls, streets with more critical locations, prisons, etc. Existing psychological-expression recognition methods can be combined with other networks. It can automatically detect various features of pedestrians in the crowd to ensure the accuracy is improved.

Based on the assumption of the consistent grey level of the optical flow method, the visual flow method cannot detect scenes or objects with changing brightness and has stricter requirements on the environment. The camera cannot rotate too fast. Therefore, psychological-expression recognition can be performed in interrogation rooms and negotiation rooms where the brightness is relatively fixed, and the target does not need to move. Psychological-expressions are based on the premise that the target suppresses their expressions, but when faced with a specific scene, the mark may have the problem of combining psychological-expressions and psychological-expressions. The work proposed by Shreve et al. [36] proposed a solution for this type of problem by using the optical flow method, making psychological-expression recognition more suitable for more stringent places such as interrogation rooms and optical flow rooms. Compared with other methods, the extracted feature dimension of the optical flow method is smaller, and it is the most viable method for real-time detection. For local binary mode improvement methods, such as pixel-by-pixel analysis methods such as LBP-TOP, the overall brightness change of the environment has little effect on it, so it can be used as a complement to the optical flow method, but its obvious disadvantage is that in the extracted feature dimension, the number is too high and the computational burden is too large for real-time detection, so it can be used as a behind-the-scenes tool for psychological-expression calibration and recognition. With the current research, after the feature dimension extracted by such methods is reduced to real time, it may be necessary to extract specific parts of the target's face, and it is necessary to minimize the occlusion of the key parts of the target to be detected. Therefore, such methods are used in it that may be more suitable for areas where the behavior and clothing of the target are strictly managed, such as detention centers or the military.

LSTM for video-type inputs has a better effect. Rather than using CNN alone, it is more appropriate to use CNN as a framework, and CNN can be combined with various methods to make the improved network recognition more effective. An LSTM differs from a CNN in that it is often used to attempt to predict performance, and computational CNN, on the other hand, is meant to identify “spatial patterns” in information and performs well on pictures and sounds. For example, the TV-L1 method extracts the optical flow image and superimposes the original image as input while using the CNN + LSTM method and then sends the extracted features to the LSTM network for psychological-expression recognition. After using the ROI method, it cooperates with the Flow Net 2.0 optical flow method to identify the visual flow of a specific area and finally enables the ROI + Revised HOOF to recognize different expressions with FACS. These two methods use other optical flow methods. Still, the main body of the TVL1+LSTM method is CNN, and the visual flow method is only used as the standard input with the original image to increase the recognition accuracy, from Tables 1–4. It can be seen that CNN, as a framework, is very inclusive and can be used in combination with a variety of methods. Therefore, it is a good tool for solving image problems. The performance comparison of CNN methods is shown graphically in Figure 3.

Figure 4 shows the community features of the proposed binary method. The improved local binary mode methods performance is shown in Figure 5 and the community features for local binary mode methods are shown in Figure 6.

But the optical flow method is essential for the environment. The requirements of the database are more stringent, and it needs to be modified on this basis before it can be applied to parts outside the database.

## 6. Conclusion

Convolution neural network and its improvement, optical flow method and its improvement, and local binary pattern and its improvement are discussed in this study. The recognition of psychological-expression information can also be improved through improvements to the convolution neural network itself. Convolution neural networks can be useful for psychological-expression recognition when they have been trained to extract visual features. After decreasing random noise, the local amplification method used in this study may magnify the psychological-expression movement such that the development trend can be perceived with the unaided eye. The optical flow method is a popular method for psychological-expression identification because it can identify small moving targets, which is ideal for detecting love. However, there are also evident issues. It is necessary to refine and optimize the algorithm in order to ensure that the brightness of the identified target remains consistent, which is sometimes difficult to do in actual applications. Optical flow, on the other hand, is a reliable method for detecting face psychological expressions. Using three planes, LBP-TOP can accurately detect videos. The update of LBP-TOP minimizes the number of redundant parameters, improves the accuracy of recognizing texture features, and can do all three at once. So, using the upgraded method of LBP for psychological-expression detection would be a good idea because it improves texture recognition.

## Figures and Tables

**Figure 1:** LBP.

**Figure 2:** LBP-TOP.

**Figure 3:** Performance comparison of CNN methods.

**Figure 4:** Community feature of proposed methods.

**Figure 5:** Performance comparisons of improved local binary mode methods.

**Figure 6:** Community Feature of local binary mode methods.

**Table 1:** Performance comparison of CNN methods.

Method	Accuracy	F1-score
CNN + LSTM	60.98	65.85
ELRCN-SE	47.15	49.52
ELRCN-TE	52.44	55.63

**Table 2:** Communities comparison of CNN methods.

Method	Modularity's	NMI
CNN + LSTM	56.63	85.63
ELRCN-SE	46.52	75.62
ELRCN-TE	53.23	80.56

**Table 3:** Performance comparison of improved local binary mode methods.

Method	Accuracy	F1-score
LBP-TOP	57.16	59.63
STLBP-IP	59.51	62.45
STLBP-IIP	62.75	66.48

**Table 4:** Performance of community extraction by local binary mode methods.

Method	Modularity's	NMI
LBP-TOP	66.63	89.24
STLBP-IP	52.63	80.54
STLBP-IIP	56.62	82.26

## Data Availability

The data shall be made available upon request.
